The article "Research Progress of Single Cell Sequencing in Lung Cancer" was published in 2021. Journal: Zhongguo Fei Ai Za Zhi.

# 单细胞测序在肺癌中的研究进展

**DOI:** 10.3779/j.issn.1009-3419.2021.102.04

**Published:** 2021-04-20

**Authors:** 孟军 俞, 金晶 谭, 敬慧 王

**Affiliations:** 1 101149 北京，北京市结核病胸部肿瘤研究所，首都医科大学附属北京胸科医院肿瘤内科 Department of Medical Oncology, Beijing Tuberculosis and Thoracic Tumor Research Institute; Beijing Chest Hospital, Capital Medical University, Beijing 101149, China; 2 101149 北京，北京市结核病胸部肿瘤研究所，首都医科大学附属北京胸科医院细胞分子生物学研究室 Department of Cellular and Molecular Biology, Beijing Tuberculosis and Thoracic Tumor Research Institute; Beijing Chest Hospital, Capital Medical University, Beijing 101149, China; 3 101149 北京，北京市结核病胸部肿瘤研究所，首都医科大学附属北京胸科医院肿瘤研究中心 Cancer Research Center, Beijing Tuberculosis and Thoracic Tumor Research Institute; Beijing Chest Hospital, Capital Medical University, Beijing 101149, China

**Keywords:** 单细胞测序, 肺肿瘤, 肿瘤异质性, 肿瘤微环境, 精准治疗, Single-cell sequencing, Lung neoplasms, Tumor heterogeneity, Tumor microenvironment, Precision treatment

## Abstract

肺癌是世界上死亡率最高的恶性肿瘤，肿瘤内部存在着明显的异质性，目前研究认为这种异质性在肺癌研究中有重要的临床意义。对于这种异质性的研究通常使用测序技术，而一般测序技术只能从整体的角度解释样本之间的差异，其分辨率不足以描绘单个细胞之间的差异。因此人们迫切希望从单细胞层面来获得肿瘤微环境中的细胞类型、状态和亚群分布以及细胞之间的通讯行为等信息。单细胞测序技术解决了这一难题。利用该技术将有助于深入了解肺癌的发生和发展机制，并发现新的诊断标记物和治疗靶点，为今后肺癌患者的精准治疗提供理论参考。本文介绍了单细胞测序技术的发展，并重点讨论了其在肺癌肿瘤异质性、肺癌肿瘤微环境、肺癌侵袭和转移以及治疗反应和耐药等方面的研究。

## Abstract (en)

Lung cancer is the malignant tumor with the highest mortality rate in the world. Heterogeneity of lung cancer, usually studied by sequencing technology, is considered to have important clinical significance in current studies. However, general sequencing technology can only explain the differences between samples integrally and its resolution is not enough to describe the differences between the individual cells. Therefore, people urgently hope to understand the cell type, state, subgroup distribution in the tumor microenvironment and the communication behavior between cells in the single cell level. Single-cell sequencing technology solves this problem. Using this technique will contribute to further understanding the mechanism of the occurrence and development of lung cancer, discovering new diagnostic markers and therapeutic targets, and providing theoretical references for the precise treatment of lung cancer patients in the future. This article reviews the progress of single-cell sequencing technology and focuses on its research on lung cancer tumor heterogeneity, tumor microenvironment, invasion and metastasis, treatment response, and drug resistance.

肺癌是世界上死亡率最高的恶性肿瘤。据最新的Cancer Statistics 2021数据显示，预计2021年美国新发肺癌占癌症新发病例的12.4%，并会导致21.7%的癌症死亡，是致死率最高的恶性肿瘤^[1]^。根据国家癌症中心2019年发布的数据，肺癌是2015年我国发病率和死亡率最高的癌症^[2]^。目前肺癌的主要治疗方式为手术、化疗、放疗、靶向和免疫治疗等。靶向治疗的出现对于有特定驱动基因突变的患者产生了良好的治疗效果，但不可避免地发生耐药和疾病进展等问题^[3, 4]^。同时，缺乏预测疗效的生物标志物和缓解率较低限制了免疫治疗的临床发展。肿瘤异质性是肿瘤治疗面临困难的重要原因。目前认为单细胞层面的研究能够获得更多的关于肿瘤异质性的有价值信息。汤富酬实验室在2009年应用单细胞RNA测序(single-cell RNA sequencing, scRNA-seq)分析单个小鼠的转录组^[5]^，使单细胞层面的分析成为可能。肺癌常常表现出瘤内基因组的显著差异性，其克隆的多样性影响了临床的诊断和治疗^[6]^。单细胞测序(single-cell sequencing, SCS)技术的应用为了解肺癌免疫微环境、发生和发展以及免疫治疗机制提供了可能^[7]^。本文将介绍单细胞测序技术的相关进展，并对其在肺癌肿瘤异质性、肿瘤微环境、侵袭和转移及治疗反应和耐药性等方面进行综述。

The article "Research Progress of Single Cell Sequencing in Lung Cancer" was published in 2021. Journal: Zhongguo Fei Ai Za Zhi.

## 1 单细胞测序技术

单细胞测序的目的是通过新一代测序技术(next generation sequencing, NGS)来识别单个细胞的基因组序列信息，并获得细胞间遗传物质和蛋白质差异的信息，从而更好地了解单个细胞在微环境中的作用^[8]^。单细胞测序还可以研究单核苷酸变异、拷贝数变异、单个细胞DNA水平的基因组结构变化、RNA水平的基因表达变化、基因融合、选择性剪接、DNA甲基化和组蛋白修饰等^[9]^。

### 1.1 单细胞测序技术的发展

单细胞测序的步骤主要包括：单细胞分离、核酸扩增、构建文库、高通量测序和数据分析。其关键是提取获得完整的有活力的靶细胞。用于单细胞分离的技术方法很多，包括梯度稀释法^[10]^、机械显微操作技术^[11]^、激光捕获显微切割技术^[12]^、荧光激活细胞分选^[13]^、免疫磁分离^[14]^、微流控平台^[15]^等。

目前常用的单细胞测序平台有SMART-seq2^[16]^、Fluidigm C1^[17]^、10X Genomics^[18]^、BD Rhapsody^[18]^等。10X是到目前为止商业化最成功的平台，在主流高影响因子的期刊上有可信的数据发表，并且都与Smart-Seq数据的结果存在比较。其优点包括高通量、低成本、操作简便、流程自动化程度高、支持文献数量多等。但对细胞总量及活性要求高，缺乏质控点及平台环境较为封闭等不足也限制了其进一步的推广。总的来说，研究者应根据自己的需求选择适合自己的单细胞测序平台。

### 1.2 单细胞测序技术的应用方向

单细胞测序主要应用于单细胞基因组测序(DNA测序)、转录组测序(RNA测序)、表观遗传测序及空间转录组测序等，它们可以揭示细胞在不同阶段的功能和不同方面的特征。

单细胞基因组测序技术将分离的单个细胞的DNA进行扩增后进行高通量测序，用于揭示细胞群体间差异和细胞进化关系。到目前为止，这种测序技术主要用于发现DNA分子中的异常^[19]^。单细胞转录组测序技术主要应用于胚胎发育、免疫系统和肿瘤多个领域，鉴定多种组织中不同类型细胞转录组特征。除了基因组本身，表观遗传修饰(特别是DNA甲基化)和不同的染色质成分在基因表达调控中也起着重要作用^[20]^。单细胞测序技术的快速发展使在单细胞水平上测量DNA甲基化成为可能。通过这些单细胞表观基因组研究，可以在单细胞分辨率下分析有关染色质修饰及其潜在调控效应的信息，能够补充单细胞DNA测序和RNA测序获得的DNA变异和RNA表达之外的数据^[21]^。

单细胞空间转录组^[22]^分析将基因的表达与组织切片的免疫组化图像进行整合，从而将组织内不同细胞的基因表达信息定位到组织的原始空间位置上去，区分哪些基因在组织内是活跃的，可以直观检测组织中不同部位基因表达的差异。目前单细胞空间转录组测序技术主要用于神经科学、生物发育和肿瘤等多个领域，为细胞功能、表型和组织微环境中位置的关系提供了重要信息。

## 2 单细胞测序在肺癌中的应用

单细胞测序技术在解析人类癌症细胞和生物复杂性方面起到了重要作用，其中许多癌症是高度异质性的，这是因为除了不同的恶性细胞亚群外，还有各种基质和免疫细胞类型。目前单细胞测序技术在黑色素瘤^[23]^、乳腺癌^[24]^、结直肠癌^[25]^等肿瘤中有了广泛的应用，对肺癌的研究也在不断深入。

### 2.1 肿瘤异质性

近年来，人们对于单个肿瘤中存在的细胞多样性有了一定的了解，但对于这种异质性如何影响肿瘤行为和临床结局仍处于萌芽阶段^[26]^。

如果能对早期肺结节的细胞类型和基因图谱有所了解，那么人们就能更好地理解早期肺癌的发生和发展的机制，做到早筛早诊早治。Lu等^[27]^使用scRNA-seq技术在单细胞水平上解析磨玻璃结节腺癌(ground glass nodules adenocarcinoma, GGN-ADC)的全面图谱，成功鉴定出肿瘤细胞、内皮细胞、T细胞等8种细胞类型。通过对GGN-ADC中细胞表型的全面分析，他们对肺癌的致癌作用有了更深刻的理解，这将有助于今后的预防和治疗。

肺癌的死亡率高和治疗预后差主要在于其异质性，为了剖析肺癌的这种异质性，Maynard等^[28]^从30例肺癌患者中，获取了49份临床活检标本，这些标本分别来自治疗前和治疗中。通过对比治疗前后肿瘤微环境所发生的变化，他们发现这些细胞展现出了极为复杂和动态的肿瘤生态系统。癌细胞的scRNA-seq能比临床常规基因检测方法发现更多的靶向癌基因。治疗后存活的癌细胞表现出肺泡细胞通路活化特征，提示治疗可诱导癌细胞向原始细胞状态转变。这表明癌细胞和肿瘤微环境会在抗癌药的作用下，变得更有可塑性。

### 2.2 肿瘤微环境

单细胞技术已被用于描述肺癌^[29]^、乳腺癌^[30]^、结直肠癌^[31]^、头颈鳞状细胞癌^[32]^等的肿瘤微环境(tumor microenvironment, TME)，包括免疫细胞和基质细胞，这是其余方法无法实现的。

肿瘤浸润性髓样细胞(tumor-infiltrating myeloid cells, TIMs)包含单核细胞、巨噬细胞、树突状细胞和嗜中性粒细胞，已成为癌症生长的关键调节剂。这些细胞可以多样化地进入多种状态，进一步促进或限制肿瘤的生长，但是人们对此知之甚少。单细胞测序可以特异性识别肿瘤微环境中某一类细胞及其对应的基因表达特征。Lavin等^[33]^利用scRNA-seq分析18个肺腺癌患者的肿瘤免疫微环境，得到了*TREM2*、*CD81*、*MARCO*、*APOE*等肿瘤浸润巨噬细胞的特征性基因。

Zilionis等^[34]^使用scRNA-seq对非小细胞肺癌(non-small cell lung cancer, NSCLC)患者的TIMs进行定位，发现了25个TIMs状态，其中大多数在患者中可被重复发现。此外，他们还对小鼠TIMs进行了分析。通过比较物种间的TIM，他们发现树突状细胞和单核细胞之间的种群结构几乎完全一致。这表明不同物种的骨髓细胞高度相似。这项研究为将来解释髓系细胞在癌症中的确切作用提供理论基础，TIMs或许可成为免疫治疗新靶标。

Guo等^[29]^采用降维聚类分析NSCLC患者的单细胞测序数据，发现一些细胞类群的T细胞耗竭特征基因表达相对较低，定义它们为预耗竭细胞，并证实“预耗竭”与耗竭T细胞比率高与肺腺癌更好的预后相关。同时，他们还观察到肿瘤调节性T细胞(regulatory T cells, Tregs)内的异质性，其特征是TNFRSF9(抗原特异性Tregs的激活标记)的双峰分布，这些激活的肿瘤Tregs的基因特征与肺腺癌的不良预后相关。研究治疗前后的T细胞表达状态，有助于识别和预测接受免疫调节剂治疗的NSCLC及其他类型肿瘤的预后。

同样，Lambrechts等^[35]^通过单细胞转录组探索了肺鳞癌基质细胞的亚群分类、基因功能、关键标志基因，共鉴定出52个基质细胞亚群，包括迄今被认为是同质的不同类型的肿瘤相关成纤维细胞、内皮细胞和肿瘤浸润免疫细胞，并发现肿瘤基质细胞基因表达的动态变化，反映了肿瘤微环境的复杂性。例如，肿瘤内皮细胞下调免疫细胞归巢途径，肿瘤CD8^+^ T细胞上调脂肪酸氧化途径。因此，肿瘤基质的独特特征可能成为新颖疗法的切入点。

The article "Research Progress of Single Cell Sequencing in Lung Cancer" was published in 2021. Journal: Zhongguo Fei Ai Za Zhi.

### 2.3 侵袭和转移

侵袭和转移代表了一个高度复杂的过程，是大多数癌症患者死亡的原因之一^[36]^。

Kim等^[37]^研究了转移性肺腺癌的单细胞转录组分析。从44例患者的正常组织或早期或转移癌的208, 506个细胞中，确定了偏离正常分化轨迹并主导转移的癌细胞亚型。在所有阶段，基质和免疫细胞的动态变化创造了促肿瘤和免疫抑制的微环境。

循环肿瘤细胞(circulating tumor cells, CTCs)是指从肿瘤原发灶或转移灶脱落进入外周血液循环系统的肿瘤细胞^[38]^。CTCs是液体活检的主要靶点，是肿瘤预后监测的重要生物标志物。研究^[39]^表明，肺癌患者CTCs数量与临床不良预后相关。基于单细胞测序技术研究肺癌患者的CTC，不仅可以发现新的CTC生物标志物，还可以在分子水平上揭示肿瘤细胞的转移机制。Ni等^[40]^通过全基因组测序观察到特征性的癌症相关的单核苷酸变异和CTC外显子组中的插入/缺失。来自单个患者的每个CTC，无论癌症亚型如何，表现出的拷贝数变异(copy number variation, CNV)具有高度一致性，表明CNV与肿瘤的转移可能相关，为今后基于CNV的肺癌诊断和治疗提供思路。

小细胞肺癌(small cell lung cancer, SCLC)因较难获得组织标本无法直接对其进行单细胞测序，通过对CTC单细胞测序或可推断SCLC进化和进展。Su等^[41]^通过对化疗期间的SCLC患者的CTC进行单细胞测序来监测体细胞突变和拷贝数变化(copy number alteration, CNA)。基于单个CTC建立的CNA评分是SCLC患者化疗后临床结局的可能预测指标。该研究结果显示，与高CNA评分(≥0)相比，低CNA评分(< 0)的患者在一线化疗后的无进展生存期和总生存期均显著延长(PFS: 212 d *vs* 110.5 d, *P*=0.004, 2; OS: 223.5 d *vs* 424 d, *P*=0.000, 6)。

### 2.4 治疗反应和耐药性

尽管采取积极的治疗措施，肺癌患者5年生存率仍只有19.8%^[42]^，一部分患者会复发，甚至发生远处转移。尽管一部分复发转移患者可以从免疫检查点抑制剂获益，但大多数患者预后很差^[43]^。人们对治疗失败的肿瘤分子和遗传基础以及患者对治疗反应的预测能力的了解仍是初级的，通过单细胞测序技术可能能够对其有更深入的了解。

Min等^[44]^分析了从人肺腺癌患者异种移植的34个单细胞中获得的转录组数据，使用基因模块G64进行聚类分析，G64模块主要由细胞周期基因组成。他们发现根据基因模块G64的上调/下调可将34个单细胞明确分为两组，同样根据G64模块的表达可以将TCGA数据库中的488例肺腺癌患者分组。G64模块的高表达可能与肺腺癌患者的不良预后相关。

Kim等^[45]^从1例肺腺癌患者的异种移植瘤中分离出34例患者来源的异种移植(patient-derived xenograft, PDX)细胞。对单个肿瘤细胞进行scRNA-seq基因表达谱分析和表达突变谱分析。存活的PDX细胞上的scRNA-seq鉴定出与抗癌药物耐药性相关的候选肿瘤细胞亚群。根据激活的*KRAS*突变和风险评分(risk scores, RS)的预后价值，表达*KRAS*^*G12D*^和高RS的PDX细胞可能是耐药的。

揭示肺癌内部肿瘤细胞的亚群分布将有助于寻找到具有抗药能力的亚群，为肺癌患者的个性化治疗提供基础，单细胞测序技术可以发现新的细胞亚群，从而研发新的靶向治疗药物。Guo等^[29]^通过对14例NSCLC患者外周血、癌及癌旁组织中的T淋巴细胞进行单细胞转录组测序，分析鉴定出肺癌T细胞群体的组成，为特异性靶向T细胞亚群的免疫治疗方法提供了新的靶标。

## 3 总结与展望

目前进行的一系列工作已经可以在细胞水平上定义异质性，单细胞转录组测序是研究人类肿瘤最先进和最广泛的一种SCS技术，迄今对恶性、免疫和基质细胞亚群以及促进侵袭和转移的细胞间相互作用具有新颖发现。通过了解肿瘤的各个亚群分布，识别肿瘤内异质性，认识肿瘤微环境的构成，为今后的临床研究和个性化治疗提供了指导方向。但是单细胞测序仍存在较多的问题有待改善，如基因组和转录组在扩增时应尽量提高覆盖率; 降低测序过程中的技术噪音; 提高单细胞的分离水平等。总的来说，单细胞测序技术的应用必将大大推动肺癌研究的进一步发展。
